The article "Multimodal Medical Image Fusion Based on Multiple Latent Low-Rank Representation" was published in 2021. Journal: Comput Math Methods Med.

# Multimodal Medical Image Fusion Based on Multiple Latent Low-Rank Representation

**DOI:** 10.1155/2021/1544955

**Published:** 2021-09-28

**Authors:** Xi-Cheng Lou, Xin Feng

**Affiliations:** School of Mechanical Engineering, Key Laboratory of Manufacturing Equipment Mechanism Design and Control of Chongqing, Chongqing Technology and Business University, Chongqing 400067, China

## Abstract

A multimodal medical image fusion algorithm based on multiple latent low-rank representation is proposed to improve imaging quality by solving fuzzy details and enhancing the display of lesions. Firstly, the proposed method decomposes the source image repeatedly using latent low-rank representation to obtain several saliency parts and one low-rank part. Secondly, the VGG-19 network identifies the low-rank part's features and generates the weight maps. Then, the fused low-rank part can be obtained by making the Hadamard product of the weight maps and the source images. Thirdly, the fused saliency parts can be obtained by selecting the max value. Finally, the fused saliency parts and low-rank part are superimposed to obtain the fused image. Experimental results show that the proposed method is superior to the traditional multimodal medical image fusion algorithms in the subjective evaluation and objective indexes.

## 1. Introduction

Medical imaging modalities are varied, each of which provides different information about organs in the body. For example, computerized tomography (CT) has excellent resolution, enabling examination of finer details in tissue, but it is weak in showing the global organ structure and pathological changes. Magnetic resonance imaging (MRI) reveals remarkable soft tissue definition with high spatial resolution, but it is limited in detecting fractures. Furthermore, anatomical imaging techniques such as CT and MRI can not reflect the body's movement information, such as metabolism. Positron emission tomography (PET) and single-photon emission computed tomography (SPECT) can visualize metabolic processes and other physiological activities, such as blood flow and regional chemical composition absorption [1]. Nevertheless, functional imaging techniques such as PET and SPECT have a low spatial resolution. In summary, it is impossible to obtain all the details of an organ from a separate imaging modality. For improving the clinical accuracy of diagnosing based on medical images, an effective method is multimodal medical image fusion, which combines multiple medical images from various modalities to improve quality and reduce redundancy of imaging.

Most medical image fusion algorithms are based on the multiscale transform (MST), which converts the source images into the transform domain and obtain the transformed coefficients through preset functions. Then, the processed coefficients can be converted to the fused image by inverse MST. According to the different decomposition methods of source images, MST can be divided into pyramid-based methods [2–4], wavelet-based methods [5–8], and multiscale geometric analysis- (MGA-) based methods [9–18]. Due to the limitation of preset functions in the MST-based algorithm, some essential features of the source images, such as edge and texture information, may not be well expressed and extracted, which significantly reduces the fusion performance. Moreover, the MST-based algorithm is usually sensitive to misregistration.

The article "Multimodal Medical Image Fusion Based on Multiple Latent Low-Rank Representation" was published in 2021. Journal: Comput Math Methods Med.

Yang and Li [19] first applied sparse representation (SR) [20] in image processing. SR decomposes the source images into several patches through a sliding window and rearranges these patches to sparse coefficient vectors, which are the linear combination of vectors in the dictionary matrix. Then, the fused image's sparse coefficient vectors can be determined through maximal *l*_1_-norm, rearrange these vectors to patches of fused image, and put these patches return to the seat can obtain the fused image. In terms of edge feature extraction, SR has certain advantages over MST. Many improved versions of SR have appeared in recent years to increase computational efficiency or improve fusion quality. Liu and Wang [21] proposed adaptive sparse representation (ASR), with seven subdictionaries trained in advance to match the patches of images categorized by the gradient. Liu et al. [22] proposed convolutional sparse representation (CSR), which does not use the sliding window to decompose the source image but applies a globe process. Liu et al. [23] proposed convolutional sparsity-based morphological component analysis (CSMCA), which simultaneously achieves multicomponent and global SR by integrating CSR and the morphological component analysis into a unified framework. However, since the SR-based algorithm's dictionary matrix cannot fully include source image data, it fails to extract the source image's detailed texture information. Some scholars applied MST [24–26] or filter [27–29] to decompose the source images. And SR can be used to fuse the low-frequency subbands. Theoretically, such methods can preserve the edge information of the image better than using SR [30] to decompose the source images. Liu et al. [31] proposed the low-rank representation (LRR), which applies the source image as the dictionary matrix, and can solve dictionary completeness. Liu and Yan [32] proposed the latent low-rank representation (LatLRR), an improved version of LRR, which can decompose the source image to saliency part, low-rank part, and noise part. Li et al. [33] proposed MDLatLRR, which integrated SR and LatLRR by using a sliding window to sample the saliency parts of LatLRR and processed the sparse coefficient vectors just like in SR-based methods. LatLRR has an extraordinary capacity for extracting texture from the image, but the ability to extract high-frequency information is not as good as MST.

The article "Multimodal Medical Image Fusion Based on Multiple Latent Low-Rank Representation" was published in 2021. Journal: Comput Math Methods Med.

Another type of image fusion method that is more widely used is with the help of weighted maps [34, 35], and deep learning-based methods are particularly suitable for generating weighted maps due to their superior feature recognition capabilities. The deep learning-based methods [36–42] have been widely used in image fusion with the development of artificial intelligence. These methods have a prominent ability to extract feature information from the image. Therefore, it is wise to use deep learning-based methods to deal with high-frequency information after image decomposition or generate the weight map as the basis of image region fusion. Wang et al. [36] applied a convolutional neural network (CNN) to generate weight maps and decompose the source images and weight maps by contrast pyramid and Laplacian pyramid, respectively, and make the Hadamard product of each decomposition layer. Finally, the fused image can be reconstructed through the contrast pyramid. Xu et al. [37] applied LatLRR to decompose source images and processed the low-rank parts by CNN and pyramid-based methods, superimposed the fused low-rank part, and fused saliency part to obtain the fused image. Liu et al. [38] applied CNN to generate weight maps and use the Laplacian pyramid and Gaussian pyramid to decompose the source images and weight maps, respectively, though the Hadamard product to obtain fused layers, and the fused image can be reconstructed through the Laplacian pyramid. Li et al. [39] applied the average filter to decompose the source images, and the fused base layer can be obtained by comparing the max absolute value of images in four convolutional layers of the VGG-19 neural network. The fused image can be obtained by superimposing the base layer and detail layer. Yin et al. [40], Tan et al. [41], and Panigrahy et al. [42] applied nonsubsampled shearlet transform (NSST) to decompose the source images and selected the fused high-frequency subbands by more firing times in the parameter-adaptive pulse coupled neural network (PAPCNN), bounded measured pulse coupled neural network (BMPCNN), and weighted parameter adaptive dual-channel pulse coupled neural network (WPADCPCNN), respectively.

As mentioned above, each method has its drawbacks and advantages. In this paper, the source images are repeatedly decomposed through LatLRR to extract the saliency parts. The fused saliency parts can be obtained by selecting the max value. After superimposing these saliency parts, the structure and edge information of the source images will be well preserved and enhance the lesion's display. Then, the VGG-19 network is used to extract features of the low-rank part, and the weight maps can be generated to be the basis of the low-rank part's activity level. The weight maps and low-rank parts then make the Hadamard product to obtain the fused low-rank part. Finally, the fused image can be obtained by superimposing the fused saliency part and fused low-rank part. The experimental results also show that the proposed method is significantly better than the comparison method regarding image information retention. The main contributions of this paper are described as follows:

1. The proposed method applies the image detail retention capability of LatLRR while fully extracting the high-frequency information of an image by iteratively decomposing the original image. It compensates for the deficiency of LatLRR and enhances the display of the lesion by superimposing saliency parts
2. The feature map of the low-rank part of the original image is extracted using the VGG-19 network and then scaled up to match the size of the original image. The weight map generated in this way can well fit the low-rank part of the original image with pixel information blockwise distributed

The rest of this paper is organized as follows.  Section 2 introduces the multiple LatLRR decomposition algorithm, Section 3 introduces the fusion rules, Section 4 describes the algorithmic structure of the proposed method, Section 5 provides a detailed discussion of the experimental results, and Section 6 concludes this paper.

The article "Multimodal Medical Image Fusion Based on Multiple Latent Low-Rank Representation" was published in 2021. Journal: Comput Math Methods Med.

## 2. Multiple Latent Low-Rank Representation

LatLRR is an improved version of LRR, whose principle is date **X** = {**x**_1_, **x**_2_, ⋯, **x**_*M*_} in space **R**^*n*^ can be represented by a linear combination of vectors in an overcomplete dictionary **D** ∈ **R**^*n*×*m*^(*n* < *m*), as

(1) $$\begin{array}{c} X=DZ, \end{array}$$

where **Z** = {**z**_1_, **z**_2_, ⋯, **z**_*M*_} is the coefficient matrix in space **R**^*m*^; it can be determined through

(2) $$\begin{array}{c} \underset{Z}{\min}{\left\|Z\right\|}_{*}\;s.t.X=DZ, \end{array}$$

where ‖·‖_∗_ denotes the nuclear norm. The idea of this algorithm is similar to that of SR, in that it finds the coefficients of an image under certain dictionary conditions. LRR using date **X** itself as the dictionary, just like equation (3), that is the reason LRR does not have the problems of dictionary training or completeness.

(3) $$\begin{array}{c} \underset{Z}{\min}{\left\|Z\right\|}_{*}\;s.t.X=XZ. \end{array}$$

The noise component **E** is added in equation (3); this is because the original purpose of creating the low-rank algorithm is to remove noise from the image. And Equation (4) is the formula of LRR.

(4) $$\begin{array}{c} \underset{Z,E}{\min}{\left\|Z\right\|}_{*}+\lambda {\left\|E\right\|}_{1,2}\;s.t.X=XZ+E, \end{array}$$

where *λ* > 0 is balance coefficient and ‖**E**‖_1,2_ denotes the *l*_1,2_-norm of **E**.

However, there are two prerequisites for using **X** itself as a dictionary. One is that the data vector of **X** must be sufficiently complete. Second, the noise of **X** must be controlled in a small range. In many practical conditions, such requirements are challenging to achieve. For this reason, the method of adding hidden items in the dictionary is proposed in [32]

(5) $$\begin{array}{c} \underset{Z}{\min}{\left\|Z\right\|}_{*}\;s.t.X_{O}=\left[X_{O},X_{H}\right]Z, \end{array}$$

where **X**_O_ denotes the known image data and **X**_*H*_ denotes the unknown hidden data. Since the dictionary contains hidden data, this improved algorithm is called the latent low-rank representation. The influence of noise is taken into account; then, we rewrite equation (5) into

(6) $$\begin{array}{c} \underset{Z,E}{\min}{\left\|Z\right\|}_{*}+\lambda {\left\|E\right\|}_{1}\;s.t.X_{O}=\left[X_{O},X_{H}\right]Z+E, \end{array}$$

where *λ* > 0 is the balance coefficient and ‖**E**‖_1_ denotes the *l*_1_-norm of **E**. Simplify equation (6) by computing the skinny singular value decomposition (SVD) of [**X**_O_, **X**_*H*_] [32], and equation (7) can be obtained.

(7) $$\begin{array}{c} \underset{Z,L,E}{\min}{\left\|Z\right\|}_{*}+{\left\|L\right\|}_{*}+\lambda {\left\|E\right\|}_{1}\;s.t.X=XZ+LX+E, \end{array}$$

where **L** denotes the saliency coefficient and **Z** denotes the low-rank coefficient. Equation (7) can be solved by the augmented Lagrange multiplier (ALM) [43]; the low-rank part and saliency part of the image could be represented as **XZ** and **LX** accordingly. The LatLRR decomposition results are shown in Figure 1. LatLRR decomposes the source image **X** to the saliency part **LX**, the low-rank part **XZ**, and the noise part **E**. **LX** contains the local structure information and saliency features or can be thought of as high-frequency information. **XZ** contains more global structure information and brightness information or can be thought of as low-frequency information. **E** denotes the'superfluous' part that LatLRR separates.

It is worth noting that in images with high spatial resolution, such as CT and MRI, detailed textures may contain essential diagnostic information. Therefore, denoising such images may filter out some critical information. In this case, a reasonable approach is to superimpose the noise part and low-rank part. Moreover, the saliency part **LX** contains most edge and structure information of the image so that the lesions may mainly reflect in the saliency part. If the low-rank part of the image is decomposed repeatedly, the saliency part will be further extracted. As shown in Figure 2, a two-layer LatLRR decomposition structure, after completing the first layer of LatLRR decomposition, the new object of LatLRR decomposition could be obtained through **X**_1_ = **XZ** + **E**, which can be further decomposed into saliency part **LX**_1_, low-rank part **X**_1_**Z**, and noise part **E**. The source images are denoted as **I**_1_ and **I**_2_. If the number of LatLRR decomposition layers is *N*, there will be *N* saliency parts {**I**_1_^*S*,*i*^}_*i*=1_^*N*^ or {**I**_2_^*S*,*i*^}_*i*=1_^*N*^ and one low-rank part **I**_1_^*L*^ or **I**_2_^*L*^ for each source image. The display of the edge and structure information will be strengthened in the new image to highlight the lesions by superimposing saliency parts. However, suppose the number *N* of LatLRR decomposition layers is blindly increased, which will reduce the efficiency of calculation. More importantly, the final fused image will display some artificial information unacceptable for medical images. In this paper, the optimal number of LatLRR decomposition layers will be determined through the experiment in Section 5.1.

The article "Multimodal Medical Image Fusion Based on Multiple Latent Low-Rank Representation" was published in 2021. Journal: Comput Math Methods Med.

## 3. Fusion Regulation

The saliency parts of the image include most high-frequency information. For multimodal medical images, the critical diagnostic information reflected by a single image is not the same. Therefore, the max-rule is applied to fuse the saliency parts of the image can preserve a single image's diagnostic information as much as possible. On the other hand, Simonyan and Zisserman [44] first applied the VGG network to extract features at different layers from images and obtain a splendid result. With the development of deep learning, the operation efficiency and precision of the VGG network have been significantly improved. As the number of LatLRR decomposition layers increases, the source image's low-rank part will contain less information. If the recognition results of VGG-19 are extracted and processed, the weight map with regional emphasis can be generated. Then, the fused low-rank part can be obtained by multiplying the weight map with the source image's low-rank part. Besides, because PET and SPECT images are in color, they need to be converted into YUV color space before fusing them with the grayscale image as MRI.

The article "Multimodal Medical Image Fusion Based on Multiple Latent Low-Rank Representation" was published in 2021. Journal: Comput Math Methods Med.

### 3.1. Fusion of Saliency Parts

Each LatLRR decomposition of the two source images will produce a saliency part of each. By adopting max-rule for all saliency parts of *N* layers of LatLRR decomposition, *N* fused significant parts can be obtained, as

(8) $$\begin{array}{c} {\left\{I_{S}^{i}\right\}}_{i=1}^{N}\left(x,y\right)=\max\left[{\left\{I_{1}^{S,i}\right\}}_{i=1}^{N}\left(x,y\right),{\left\{I_{2}^{S,i}\right\}}_{i=1}^{N}\left(x,y\right)\right], \end{array}$$

where {**I**_*S*_^*i*^}_*i*=1_^*N*^(*x*, *y*) denote the position (*x*, *y*) of the *i*th layer saliency part of fused image {**I**_*S*_^*i*^}_*i*=1_^*N*^, so as {**I**_1_^*S*,*i*^}_*i*=1_^*N*^(*x*, *y*) and {**I**_2_^*S*,*i*^}_*i*=1_^*N*^(*x*, *y*). The final fused saliency part can be calculated by

(9) $$\begin{array}{c} I_{S}=\overset{N}{\underset{i=1}{\sum }}I_{S}^{i}. \end{array}$$

### 3.2. Fusion of Low-Rank Parts

VGG-19 is a convolutional neural network that is 19 layers deep, including 16 convolutional layers and 3 fully connected layers. Its structure is shown in Figure 3. Each convolutional layer is denoted as conv‘size of the filter'-‘number of such filters,' and max-pooling layers have 2 × 2 filter with the stride of 2. The information of the low-rank part of the image after multiple LatLRR decompositions is relatively fuzzy and presents a regional-like distribution. According to this feature, the feature maps extracted from the fifth convolution layer of VGG-19 can match the low-rank part of the image's information distribution state after amplification.

For low-rank parts **I**_1_^*L*^ and **I**_2_^*L*^, {*ϕ*_1_^*m*^}_*m*=1_^512^ and {*ϕ*_2_^*m*^}_*m*=1_^512^ denote the feature maps extracted from the fifth convolutional layer of VGG-19. As shown in Figure 3, the 5th convolutional layer is conv3-512, so there are 512 feature maps of each low-rank part. Moreover, because of max-pooling layers, these feature maps are only (0.5)^5^ the size of the source image. According to [39], let {*ϕ*_*k*_^*m*^}_*m*=1_^512^(*x*, *y*) denote the (*x*, *y*) position of the *k*th low-rank part's feature maps, where *k* ∈ {1, 2}. The *l*_1_-norm of {*ϕ*_*k*_^*m*^}_*m*=1_^512^(*x*, *y*) could be the activity level measure of the low-rank part. So, the activity level map **C**_*k*_ can be calculated by

(10) $$\begin{array}{c} C_{k}\left(x,y\right)={\left\|{\left\{\phi_{k}^{m}\right\}}_{m=1}^{512}\left(x,y\right)\right\|}_{1}. \end{array}$$

Then, the initial weight map ${\hat{W}}_{k}$ can be obtained by

(11) $$\begin{array}{c} {\hat{W}}_{k}\left(x,y\right)=\frac{C_{k}\left(x,y\right)}{C_{1}\left(x,y\right)+C_{2}\left(x,y\right)}. \end{array}$$

As feature maps are only (0.5)^5^, the size of the source image, so the initial weight map ${\hat{W}}_{k}$, which is generated by feature maps, is (0.5)^5^ the size of the source image too. For matching the size of the source image, ${\hat{W}}_{k}$ need the upsampling procedure as

(12) $$\begin{array}{c} W_{k}\left(x,y\right)={\hat{W}}_{k}\left(x+p,y+q\right)\;p,q\in \left\{1,2,\cdots ,15\right\}. \end{array}$$

The fused low-rank part **I**_*L*_ can be calculated by

(13) $$\begin{array}{c} I_{L}=W_{1}\circ I_{1}^{L}+W_{2}\circ I_{2}^{L}, \end{array}$$

where ∘ denotes the Hadamard product.

The article "Multimodal Medical Image Fusion Based on Multiple Latent Low-Rank Representation" was published in 2021. Journal: Comput Math Methods Med.

### 3.3. YUV Color Space

For color images such as SPECT and PET, Yin et al. [40] proposed a YUV space to solve color and grayscale images' fusion problems. The color image is first converted to YUV space and decomposed into one luminance component, ‘Y' and two chrominance components, ‘U' and ‘V.' Then, the ‘Y' component of the color image can be fused with the grayscale image by the proposed method. The final fused image can be obtained through transforming the fused component ‘Y' and other two chrominance components ‘U' and ‘V' from YUV space to the RGB space, as shown in Figure 4.

### 3.4. Reconstruction

Superimpose the fused low-rank part **I**_*L*_ and fused saliency part **I**_*S*_ to reconstruct fused image **I**_*F*_ as

(14) $$\begin{array}{c} I_{F}=I_{S}+I_{L}. \end{array}$$

## 4. Structure of Algorithm

Source images **I**_1_ and **I**_2_ have been registered, the algorithm framework in this paper as showed in Figure 5.

The main steps of the proposed method are summarized as Algorithm 1.

## 5. Experiment

Five sets of registered multimodal medical images collected from The Whole Brain Atlas [45] are used to verify the effectiveness of the proposed method, as shown in Figure 6. Figures 6(a) and 6(b) are the first set of images from a 55-year-old patient with multiple embolic infarctions; Figures 6(c) and 6(d) are the second set of images from a 31-year-old man with cerebral toxoplasmosis; Figures 6(e) and 6(f) are the third set of images from a 51-year-old patient with anaplastic astrocytoma; Figures 6(g) and 6(h) are the fourth set of images from a 70-year-old patient with mild Alzheimer's disease; Figures 6(i) and 6(j) are the fifth set of images from a 36-year-old patient with infectious disease due to HIV positive.

All the experiments in this paper are conducted on a PC equipped Intel(R) Xeon(R) CPU E3-1231 v3 (3.40 GHz) and 16 GB RAM. The software environment is MATLAB R2019b installed on Win 10 64-bit operating system.

### 5.1. Parametric Experiment

In order to determine the decomposition layers of LatLRR in this paper, five sets of images in Figure 6 were fused by the proposed method. The results are objectively evaluated by four fusion image evaluation indexes: fusion metric-based on Tsallis entropy (*Q*_TE_) [46], gradient-based fusion performance (*Q*_G_) [47], image structural similarity metric (*Q*_C_) [48], and human perception inspired fusion metric (*Q*_CB_) [49]. *Q*_TE_ is a divergence measure of the degree of dependence between two discrete random variables, and it calculates information from the source images is transferred to the fused image. Therefore, the larger the *Q*_TE_ value, the better the fusion effect. *Q*_G_ uses the Sobel edge operator to calculate the intensity and direction information of the edges in the source image and the fused image. The larger the *Q*_G_ value is, the richer the edge information of the fused image is. *Q*_C_ is used to measure the preservation degree of structure of the fused image, so it calculates how much of the salient information in each source image has been transferred into the fused image. The larger the *Q*_C_ is, the better the structure of the source images is preserved. The calculation process of *Q*_CB_ is complex and consists of five steps: contrast sensitivity filtering, local contrast computation, contrast preservation calculation, saliency map generation, and global quality map computation. *Q*_CB_ takes the mean value of the global quality map. The larger the *Q*_CB_ value is, the richer the contrast information of the fused image is.

The article "Multimodal Medical Image Fusion Based on Multiple Latent Low-Rank Representation" was published in 2021. Journal: Comput Math Methods Med.

The test decomposition layers of LatLRR are set from 1 to 4. Parameter experimental results of indexes of four sets of images are shown in Figures 7(a)–7(d). It can be observed that as the number of LatLRR decomposition layers increases, not all indexes show a uniform trend. The value of *Q*_TE_ increased with the increase of decomposition layers, while *Q*_CB_ are optimal in the case of one-level decomposition. As for *Q*_G_ and *Q*_C_, the changing trend is related to the image set. It is reasonable because the more decomposition layers, the image background information contained in the low-rank part will be fuzzier and more contained in the saliency part. The max-rule selects the saliency part of the fused image, so the background information of the source images may also be strengthened in the fused image, enhancing the appearance of the lesion. If the greater the amount of information, the larger the *Q*_TE_ value will be. However, strengthening image background information will weaken the boundary observation and reduce the image contrast, undoubtedly leading to a lower *Q*_CB_. Medical image fusion aims to show the information of lesions in the fused image, so the *Q*_TE_ is more impotent than the other three indexes. It can be seen from Figure 7(a) that *Q*_TE_ of two decomposition layers is significantly improved than that of one decomposition layer. Still, the more decomposition layers could not considerably improve the *Q*_TE_.

The article "Multimodal Medical Image Fusion Based on Multiple Latent Low-Rank Representation" was published in 2021. Journal: Comput Math Methods Med.

Besides, as Figure 8 shows, it can be seen that with the increase of the number of LatLRR decomposition layers, the artifact around the object will be aggravated in several sets of images. In order to improve the image fusion quality, the lesion in the fused image should be highlighted as much as possible, and artifacts should be strictly controlled. Therefore, the decomposition layer of LatLRR in this paper is set as two.

### 5.2. Contrast Experiment

Nine typical multimodal medical image fusion methods are selected to compare with the proposed method: four sorts of SR-based methods, CSR [22], ASR [21], CSMCA [23], and MDLatLRR [33]; three sorts of deep learning-based algorithm, CNN [36], VGG-19 [39], and BMPCNN [41]; and two sorts of MST integrated SR methods are nonsubsampled contourlet transform (NSCT) combined with SR (NSCT_SR) [24] and Laplacian pyramid (LP) combined with SR (LP_SR) [24]. The MST decomposition level is set to 4.

Figure 9 shows the fusion results of the first set images, Figures 9(a) and 9(b) are the source images. It can be seen from Figure 9(l) of the proposed method, both the brain tissue texture in the green box and the lesion edge in the red box are the clearest from other fusion methods. Besides, the pixel consistency of bone in the proposed method is the best.  Figure 10 shows the fusion results of the second set images; Figures 10(a) and 10(b) are the source images. As can be seen in Figure 10(l), the pixel consistency of the skeletal structure of the fused images is the best, and the widening of the brain tissue sulcus in the green box, as well as the calcified lesions and edema in the red box, are also clearly visible.  Figure 11 shows the fusion results of the second set images; Figures 11(a) and 11(b) are the source images. In Figure 11(l) of the proposed method, the boundary of the metabolic abnormality in the red box is the clearest, and the chromatic aberration is most consistent with Figure 11(b). The texture information in the green box is also clearly visible.  Figure 12 shows the fusion results of the third set images; Figures 12(a) and 12(b) are the source images. In Figure 12(l) of the proposed method, the boundary of the metabolic abnormality in the red box is the most distinct, and the texture in the green box also holds the best. Besides, in this set of images, some fusion methods appear serious color distortion, as can be seen in Figures 12(c), 12(d), and 12(j), the color rendering of the proposed method is closest to the source image.  Figure 13 shows the fusion results of the fourth set images, Figures 13(a) and 13(b) are the source images. Compared with Figure 13(b), the graphic structure of metabolic abnormalities (red box) in other fusion methods has been deformed to a certain extent. The structure is kept intact in the proposed method, and the chromatic aberration is most consistent with the source image.

The article "Multimodal Medical Image Fusion Based on Multiple Latent Low-Rank Representation" was published in 2021. Journal: Comput Math Methods Med.

All the fusion images are evaluated by four indexes introduced in Section 5.1. As shown in Tables 1–5, in all sets of images, the proposed method leads in *Q*_TE_, especially in the first set of images, the lead is more than 30 percent. It means that the proposed method is superior to other methods in the information conversion of source images. Moreover, for the first set and the fourth set of images, the proposed method also leads in the *Q*_C_. And it indicates that the proposed method can retain the structure of the source images better than other methods. On the other hand, the proposed method has no advantage or even a considerable gap over the best-performing method in terms of the other two indicators. As mentioned in Section 5.1, *Q*_G_ and *Q*_CB_ are mainly used to measure the degree to which the fused image retains the edge information of the source images. *Q*_G_, in particular, is directly affected by the gradient of the fused image. As shown in Figure 12(c), the color of the CSR fusion image is seriously distorted, and the white area in the middle of the image has apparent artifacts, which is unacceptable for brain images. However, the color distortion and artifacts bring to the fused image that the ‘border' does not initially exist and will undoubtedly increase the image structure's gradient value and complexity. That is why *Q*_G_ and *Q*_CB_ of CSR show undeniable advantages in the contrast experiment of third set images. *Q*_TE_ measures the degree to which the fusion image retains the information of the source images, and the distortion of image structure or color will lower this index. Image artifacts and structural distortions may mislead medical professionals, so it is not advisable to blindly pursue high image structure indexes. The proposed method has obvious advantages in the *Q*_TE_ index, and the degree of color distortion and artifact in the fused images is minimal. It is crucial for medical images. Because artifacts in brain images can sometimes look very similar to lesions, false lesions in images can directly affect the judgment of medical professionals. In addition, SPECT and PET show metabolic abnormalities through chromatic aberration. If significant color distortions appear in the image, it will cause deviation from the real. Based on the above analysis, the proposed method is effective.

The article "Multimodal Medical Image Fusion Based on Multiple Latent Low-Rank Representation" was published in 2021. Journal: Comput Math Methods Med.

## 6. Conclusion

In this paper, a multimodal medical image fusion method based on multiple latent low-rank representation is proposed. Experimental results show that the proposed method has advantages in preserving edge features and texture details and leads to objective evaluation indexes compared with other fusion algorithms. The proposed method can enhance the observer's ability to identify the lesions and contribute to practical applications such as diagnosis, treatment planning, and surgical navigation. On the other hand, the proposed method also has some drawbacks. The highlight of lesions is based on multilayer LatLRR decomposition, but with the increase of the number of decomposition layers, artifacts will become more evident. Besides, the more layers decomposed by LatLRR, the less information of the low-rank part of the source image, and the greater the error of VGG-19 network recognition. The next stage should focus on eliminating artifacts as much as possible in the case of multilayer LatLRR decomposition and improve the fusion quality of low-rank parts of source images.

## Figures and Tables

**Figure 1:** LatLRR decomposition diagram.

**Figure 2:** Two-layer LatLRR decomposition diagram.

**Figure 3:** The procedure of low-rank part fusion.

**Figure 4:** Schematic of the grayscale and color image.

**Figure 5:** Algorithm framework.

**Figure 6:** Five sets of multimodal medical images for the experiment. (a) MR-PD. (b) CT. (c) MR-T1. (d) CT. (e) MR-T2. (f) SPECT-Tl. (g) MR-T2. (h) PET-FDG. (i) MR-T2. (j) SPECT-Tc.

**Figure 7:** Parametric experimental results. (a) *Q*_TE_ of five sets of images. (b) *Q*_G_ of five sets of images. (c) *Q*_C_ of five sets of images. (d) *Q*_CB_ of five sets of images.

**Figure 8:** The fusion result of each LatLRR decomposition level. (a) 1 layer. (b) 2 layers. (c) 3 layers. (d) 4 layers. (e) 1 layer. (f) 2 layers. (g) 3 layers. (h) 4 layers. (i) 1 layer. (j) 2 layers. (k) 3 layers. (l) 4 layers.

**Figure 9:** Comparison of the fusion results in the first set images. (a) MR-PD. (b) CT. (c) CSR. (d) ASR. (e) CSMCA. (f) CNN. (g) BMPCNN. (h) MDLatLRR. (i) VGG-19. (j) NSCT_SR. (k) LP_SR. (l) Proposed method.

**Figure 10:** Comparison of the fusion results in the first set images. (a) MR-T1. (b) CT. (c) CSR. (d) ASR. (e) CSMCA. (f) CNN. (g) BMPCNN. (h) MDLatLRR. (i) VGG-19. (j) NSCT_SR. (k) LP_SR. (l) Proposed method.

**Figure 11:** Comparison of the fusion results in the second set images. (a) MR-T2. (b) SPECT-T1. (c) CSR. (d) ASR. (e) CSMCA. (f) CNN. (g) BMPCNN. (h) MDLatLRR. (i) VGG-19. (j) NSCT_SR. (k) LP_SR. (l) Proposed method.

The article "Multimodal Medical Image Fusion Based on Multiple Latent Low-Rank Representation" was published in 2021. Journal: Comput Math Methods Med.

**Figure 12:** Comparison of the fusion results in the third set images. (a) MR-T2. (b) PET-FDG. (c) CSR. (d) ASR. (e) CSMCA. (f) CNN. (g) BMPCNN. (h) MDLatLRR. (i) VGG-19. (j) NSCT_SR. (k) LP_SR. (l) Proposed method.

**Figure 13:** Comparison of the fusion results in the fourth set images. (a) MR-T2. (b) SPECT-Tc. (c) CSR. (d) ASR. (e) CSMCA. (f) CNN. (g) BMPCNN. (h) MDLatLRR. (i) VGG-19. (j) NSCT_SR. (k) LP_SR. (l) Proposed method.

**Algorithm 1:** Proposed image fusion algorithm.

**Table 1:** Objective evaluation of fusion methods in the first set of images.

Fusion method	*Q*_TE_	*Q*_G_	*Q*_C_	*Q*_CB_	*t*/*s*
Proposed method	*0.4359*	0.5145	*0.6436*	0.5036	158.7860
CSR	0.3096	0.6608	0.5621	*0.7137*	135.2650
ASR	0.2976	*0.6700*	0.6121	0.6622	210.1220
CSMCA	0.2945	0.5830	0.5587	0.6103	372.3040
CNN	0.3247	0.6267	0.5560	0.5916	32.7860
BMPCNN	0.3058	0.5554	0.5828	0.5943	67.0890
MDLatLRR	0.2882	0.6527	0.6077	0.6784	69.0270
VGG-19	0.2835	0.5104	0.5569	0.6273	7.4480
NSCT_SR	0.2953	0.6243	0.5895	0.6353	7.4890
LP_SR	0.2948	0.6560	0.5734	0.6588	*0.3380*

**Table 2:** Objective evaluation of fusion methods in the second set of images.

Fusion method	*Q*_TE_	*Q*_G_	*Q*_C_	*Q*_CB_	*t*/*s*
Proposed method	*0.4495*	0.5647	0.6995	0.6061	50.6440
CSR	0.3911	0.6363	0.7000	*0.7454*	33.1950
ASR	0.3595	*0.7122*	*0.7532*	0.7328	64.9900
CSMCA	0.3491	0.6315	0.7090	0.6974	78.8380
CNN	0.4131	0.4757	0.6533	0.5848	13.8630
BMPCNN	0.3726	0.5354	0.6918	0.6210	15.7120
MDLatLRR	0.3657	0.6516	0.7108	0.7357	21.1340
VGG-19	0.4211	0.4030	0.6457	0.3627	5.1570
NSCT_SR	0.3725	0.5514	0.6886	0.6389	2.2760
LP_SR	0.3582	0.6025	0.6741	0.6521	*0.2210*

**Table 3:** Objective evaluation of fusion methods in the third set of images.

Fusion method	*Q*_TE_	*Q*_G_	*Q*_C_	*Q*_CB_	*t*/*s*
Proposed method	*0.7297*	0.6602	0.6249	0.4645	233.0850
CSR	0.5025	*0.8111*	0.7920	*0.7010*	130.2410
ASR	0.4632	0.7901	0.7755	0.6611	188.6130
CSMCA	0.4576	0.7319	0.6790	0.5979	390.8500
CNN	0.7183	0.7822	0.7530	0.4966	38.6490
BMPCNN	0.3832	0.7900	*0.8470*	0.6505	75.5030
MDLatLRR	0.4303	0.7755	0.7298	0.6416	73.5810
VGG-19	0.4828	0.7026	0.6891	0.6179	7.8900
NSCT_SR	0.4659	0.8054	0.8200	0.6757	9.2580
LP_SR	0.5044	0.7994	0.8120	0.5991	*0.5030*

**Table 4:** Objective evaluation of fusion methods in the fourth set of images.

Fusion method	*Q*_TE_	*Q*_G_	*Q*_C_	*Q*_CB_	*t*/*s*
Proposed method	*0.6267*	0.5968	*0.6416*	0.4832	163.4530
CSR	0.5041	*0.8026*	0.6380	*0.7370*	149.6120
ASR	0.4431	0.7291	0.6231	0.6573	192.5610
CSMCA	0.4383	0.6821	0.6355	0.6141	344.2190
CNN	0.4197	0.6749	0.5585	0.6446	33.4460
BMPCNN	0.3437	0.5930	0.6328	0.5226	71.7970
MDLatLRR	0.4270	0.6752	0.6056	0.6567	61.6160
VGG-19	0.4730	0.6605	0.5722	0.6353	7.6620
NSCT_SR	0.4529	0.6827	0.6386	0.6001	7.5950
LP_SR	0.4457	0.6734	0.5938	0.5764	*0.3240*

The article "Multimodal Medical Image Fusion Based on Multiple Latent Low-Rank Representation" was published in 2021. Journal: Comput Math Methods Med.

**Table 5:** Objective evaluation of fusion methods in the fifth set of images.

Fusion method	*Q*_TE_	*Q*_G_	*Q*_C_	*Q*_CB_	*t*/*s*
Proposed method	*0.5260*	0.6594	0.6234	0.6005	46.2110
CSR	0.5175	*0.8783*	*0.8793*	*0.8374*	22.4600
ASR	0.4639	0.7902	0.7986	0.6573	53.9060
CSMCA	0.4808	0.7908	0.8237	0.7346	76.9750
CNN	0.5186	0.7668	0.8170	0.4144	11.8690
BMPCNN	0.3632	0.7289	0.8196	0.7099	14.8240
MDLatLRR	0.4591	0.7905	0.8180	0.7464	17.9870
VGG-19	0.4947	0.6974	0.6851	0.6797	5.1760
NSCT_SR	0.4962	0.7658	0.7943	0.9358	2.2660
LP_SR	0.5083	0.7843	0.8435	0.6496	*0.2280*

## Data Availability

The data supporting the study are obtained from K. A. Johnson and J. A. Becker, *The Whole Brain Atlas*, 2021. URL: http://www.med.harvard.edu/aanlib/, (accessed 12 May 2021).
